# Recombinant *Pvs*48/45 Antigen Expressed in *E*. *coli* Generates Antibodies that Block Malaria Transmission in *Anopheles albimanus* Mosquitoes

This article has been retracted.

**DOI:** 10.1371/journal.pone.0119335

**Published:** 2015-03-16

**Authors:** Myriam Arévalo-Herrera, Andrés F. Vallejo, Kelly Rubiano, Yezid Solarte, Catherin Marin, Angélica Castellanos, Nora Céspedes, Sócrates Herrera

**Affiliations:** 1 Malaria Vaccine and Drug Development Center, Cali, Colombia; 2 Caucaseco Scientific Research Center, Cali, Colombia; 3 School of Health, Universidad del Valle, Cali, Colombia; 4 Primates Center Foundation, Cali, Colombia; Ehime University, JAPAN

## Abstract

Transmission of malaria parasites from humans to *Anopheles* mosquitoes can be inhibited by specific antibodies elicited during malaria infection, which target surface *Plasmodium* gametocyte/gamete proteins. Some of these proteins may have potential for vaccine development. *Pvs*48/45 is a *P*. *vivax* gametocyte surface antigen orthologous to *Pfs*48/45, which may play a role during parasite fertilization and thus has potential for transmission blocking (TB) activity. Here we describe the expression of a recombinant *Pvs*48/45 protein expressed in *Escherichia coli* as a ∼60kDa construct which we tested for antigenicity using human sera and for its immunogenicity and transmission blocking activity of specific anti-mouse and anti-monkey *Pvs*48/45 antibodies. The protein reacted with sera of individuals from malaria-endemic areas and in addition induced specific IgG antibody responses in BALB/c mice and *Aotus l*. *griseimembra* monkeys. Sera from both immunized animal species recognized native *P*. *vivax* protein in Western blot (WB) and immunofluorescence assays. Moreover, sera from immunized mice and monkeys produced significant inhibition of parasite transmission to *An*. *Albimanus* mosquitoes as shown by membrane feeding assays. Results indicate the presence of reactive epitopes in the *Pvs*48/45 recombinant product that induce antibodies with TB activity. Further testing of this protein is ongoing to determine its vaccine potential.

## Introduction

Malaria is transmitted in ∼106 countries in tropical and subtropical regions of the world where over 207 million clinical cases and 1 million deaths were reported in 2013 [1]. This represents a huge social and economic burden worldwide. Individuals that are continuously exposed to malaria infection in endemic regions eventually develop clinical immunity that protects them from severe disease, complications, and death; however, sterile immunity is never achieved under natural conditions [2–4]. These individuals also develop immune responses that reduce or completely block parasite transmission from humans to the mosquito vector in what has been called transmission blocking (TB) immunity [5]. It has been experimentally demonstrated that specific antibodies targeting *Plasmodium* antigens which are expressed on gametocytes, zygote, gametes and ookinete stages can block parasite transmission from a variety of malaria animal hosts, including humans and non-human primates, to mosquitoes [6–11].

Therefore TB immune mechanism may represent an important method to prevent human malaria transmission and may eventually contribute to malaria elimination. However, the malaria TB process appears to be complex and depends on multiple factors such as target antigens, time of antigen expression, antibody concentration, and in some cases, on complement activation [12–14]. In *P*. *falciparum*, as in other species, several gametocyte antigens, i.e., *Pfs*230 and *Pfs*48/45, as well as oocyst/ookinete antigens, i.e., *Pfs*25 and *Pfs*28, which have been identified as potential TB vaccine candidates, have been expressed as recombinant proteins [8,15–19]. However, efforts to express some of these proteins with their proper conformation to induce antibodies with TB capacity have been hampered by the presence of the high number of cysteine residues that usually lead to complex protein structures. Functional protein domains appear to contain conformational epitopes that are recognized by antibodies capable of blocking the corresponding functional activities [20]. It has been shown in *ex-vivo* assays that there is a strong correlation between antibody titers to *Pfs*48/45 present in sera of individuals from malaria-endemic areas and the TB activity displayed [21,22]. The demonstration that *Pfs*48/45 is required in the parasite fertilization process as well as its presence on the gametocyte surface membrane [23] which may lead to potential boosting of anti-*Pvs*48/45 antibodies during natural infections have raised interest in this protein as a TB vaccine candidate.

*Both P*. *vivax Pvs*25 and *Pvs*28 proteins are expressed after parasite fertilization in the mosquito midgut [24] and both have been produced as recombinant proteins and tested in preclinical studies [8,19,25–27]. *Pvs*25 has been further assessed in clinical trials [28,29]. Studies with *P*. *vivax* pre-fertilization antigens are limited due to the difficulty of producing these proteins with proper structural conformation and in sufficient amounts [30]. Additionally, malarial proteins contain multiple potential glycosylation sites whereas prokaryotic expression systems such as *E*. *coli* lack N-linked glycosylation machinery and use periplasmic oxidoreductases for correct disulphide bond formation in the periplasmic space [31]. Despite the considerable advantages of the *E*. *coli* system for recombinant protein production, there are major technical hurdles like the formation of inclusion bodies as a consequence of high-level protein production with low amounts of active protein contained in insoluble aggregates in the cytoplasm [32]. This study had three aims related to *Pvs*48/45: First, to optimize its expression using full-length codon harmonization. Second, to assess its antigenicity in humans and its immunogenicity in BALB/c mice, a rodent species commonly used in immunological studies, and in *Aotus lemurinus griseimembra* monkeys, the non-human primate species most susceptible to human malaria parasites infection [33]; third, to assess the functional TB capacity of the elicited antibodies.

## Material and Methods

### Ethics Statement

This study was carried out in accordance with institutional guidelines. Human sera for antigenicity studies were collected as part of a malaria epidemiology study in the context of an International Center of Excellence for Malaria Research (ICEMR) program. The protocol was reviewed and approved by NIH (DMID No. 11-0028) and the IRB of Malaria Vaccine and Drug Development Center-MVDC (Cali-Colombia) (Code 004-2010). Written informed consent (IC) was obtained from each volunteer at enrollment and information obtained from the participants was managed on principles of confidentiality. Ethical clearance to draw blood samples from *P*. *vivax* infected blood was obtained by prior written IC which was previously approved by the Ethical Committee of the MVDC IRB (CECIV). Immediately after blood donation, volunteers were provided with the antimalarial treatment recommended by the Colombian Ministry of Health (chloroquine/primaquine).

Animal studies were performed according to the national animal protection status from Colombia (Law 84/98) and the Guidelines of the National Institutes of Health for the Care and Use of Laboratory Animals [34]. The protocol was approved by the Committee for Animal Ethics of MVDC.

#### Aotus monkeys housing and husbandry

New World *Aotus l*. *griseimembra* monkeys, originally from the northern forests of Colombia, are considered to be one of the non-human primate species most susceptible to human malaria infections [33]. Adult animals were kept in captivity at the Fundación Centro de Primates-FUCEP (Cali, Colombia) in single cages of ∼1x1x1meter/monkey, provided with hiding niches and maintained in natural temperature conditions at an annual average of ∼25°C. Animals were fed with fresh tropical fruits and vegetables, commercially available pet chow, and vitamin supplement.

*Aotus* selected for this study were subjected to liver and kidney functional tests (Creatinine: <0.6 mg/dL, ALT < 135 U/L, AST <250 U/L) as well as hemoglobin (13–15 g/dL) and hematocrit (40–50%) measurements. Clinical and laboratory evaluation was made before immunization and after the end of the study. If loss of appetite or weakness were observed, further clinical testing and evaluation was performed, such hematology and chemical to ensure healthy conditions. An experienced veterinarian and technicians were in charge of animal handling which did not require anesthesia. The endpoints considered for the monkeys were decrease of body weight, lack of appetite, skin`s lesions in the immunization site due to the adjuvant, corporal temperature (>38°C), dehydration test (>10%), low levels of Haematocrit/hemoglobin (Hto: 50% and Hb: 9g/dL) and changes on the biochemistry parameters (Renal and Hepatic function). None of the animals died during the course of the research. After the end of the study and healthy conditions verification, monkeys were transferred to a rest or reproduction modules where they are kept alive with food and water supply until their natural death.

### Protein Production

#### Sequence Alignment

*Pvs*48/45 gene sequence data and gene expression profiles were analyzed using the resources provided by the PlasmoDB website (http://PlasmoDB.org; accession no. PVX_083235). Identification of functional domains from the amino acid sequence was performed on servers SMART (SimpleModular Architecture Research Tools) and Pfam. Homologous sequences from *P*. *falciparum (PF3D7_1346700)*, *P*. *knowlesi (PKH_120750)*, *P*. *berghei (PBANKA_135960)*, *P*. *chabaudi (PCHAS_136420)* and *P*. *yoelii (PYYM_1361700)* were used to construct alignments and determine sequence similarity between species.

#### Codon Harmonization

The *P*. *vivax Pvs*48/45 gene was harmonized for production in *E*. *coli* using the codon harmonization algorithm in the EuGene software v0.92 [35]. The harmonized *Pvs*48/45 sequence was analyzed to optimize the codon context and eliminate repeat regions, thereby avoiding hidden stop codons and possible intermediate Shine Dalgarno sequences [35]. In addition, the GPI anchor was removed and restriction sites were added to the 5’ and 3’ regions for in-frame cloning. The final gene was analyzed in Bioedit sequence alignment editor version 7.0.5.3 [36] to ensure the correct read frame of the tagged fusion protein.

#### Cloning, Expression and Purification of *Pvs*48/45 Protein

The synthetic gene (IDT Technologies) and the expression plasmid pET32a were simultaneously digested with Alu I (Fermentas) and BamHI (Fermentas) and separated by agarose gel electrophoresis. Gel bands corresponding to the *Pvs*48/45 insert and pET32a expression vector were purified using a high pure, DNA clean-up protocol. Ligation was performed in a 3:1 vector/insert ratio using a Rapid DNA Ligation Kit (Fermentas) according to the manufacturer’s instructions. The product was transformed into competent Novablue *E*. *coli* cells (Novagen) and plated out for primary selection. Positive clones were selected using PCR. *E*. *coli* Origami 2 cells were used for protein expression. Overnight cultures were diluted 20-fold and grown at 25°C until an OD 600nm of 0.4. A final concentration of 0.1 mM Isopropyl β-D-thiogalactopyranoside (IPTG) was added for overnight induction of protein expression. Cultures were then centrifuged at 4000 rpm for 15 min and the pellets were lysed using RIPA buffer. The soluble fraction obtained was purified by affinity chromatography using immobilized metal ion affinity chromatography with a histidine select cobalt resin (Pierce) following the manufacturer’s instructions. The protein was refolded by dialysis with a gradient of increasing concentration of arginine-based buffer (arginine 0.5 M /TBS pH: 7.4). Endotoxins were removed using High Capacity Endotoxin Removal Resin (Pierce, USA). Fractions were analyzed by SDS-PAGE and pooled for identification analysis.

### Protein Characterization

#### Mass Analysis

Identity of the *Pvs*48/45 recombinant protein was analyzed by mass spectrometry (LC-MS/MS). The target protein solution was subjected to in-solution alkylation/tryptic digestion followed by LC-MS/MS analysis as described previously [37]. Briefly, the protein was digested overnight at 37°C with proteomics-grade trypsin (20 ng/μL) and the tryptic peptides were purified by reverse-phase chromatography using PepClean C-18 spin columns according to the manufacturer’s instructions (Pierce). The mixture of peptides was then subjected to electrospray mass analysis on an ion triple quadrupole trap LC-MS/MS with 3200 Q TRAP (Applied Biosystems, Foster City, CA). Peptide mass spectra obtained from the digested protein were searched against protein mass fingerprinting databases using MASCOT and Scaffold software.

#### Immunoblot Analysis

Protein fractions separated by sodium dodecyl sulfate polyacrylamide gel electrophoresis (SDS-PAGE) were transferred to a nitrocellulose membrane according to the method described by Blake [38]. The membrane was blocked with Tris Buffered Saline with Tween 20 (TBST) 0.5% milk at room temperature for 2 hours, washed 5 times with TBST for 5 minutes, and cut into strips that were incubated for 1 hour with anti-His antibody (Sigma-Aldrich) at 1:10,000 or with a positive control, which consisted of a pool of hyperimmune sera from *P*. *vivax-*immune primates at 1:50. Strips were then incubated for 1 h with either alkaline phosphatase-conjugated anti-mouse IgG or anti-human IgG antibodies respectively (Sigma-Aldrich) at a dilution of 1:10,000 and were then washed as before. Finally, formation of immune complexes in the membrane was assessed visually by adding TMB or NBT-BCIP substrates (Sigma Aldrich) accordingly.

#### Analysis of Human Sera

Antigenicity of the *Pvs*48/45 recombinant product was assessed with 30 human sera from individuals naturally exposed to *P*. *vivax* in endemic areas of Colombia with different malaria transmission intensity as well as *P*. *vivax* and *P*. *falciparum* distribution. Tierralta in the Caribbean region displayed higher transmission intensity than Tumaco, Buenaventura and Quibdó in the Pacific region. Additionally, Tierralta and Buenaventura displayed higher *P*. *vivax* transmission than Tumaco and Quibdo where *P*. *falciparum* was predominant [39]. The presence of antibodies to *Pvs*48/45 was determined by enzyme-linked immunosorbent assay test (ELISA) as described below. In order to ascertain previous exposure of serum-donors to *P*. *vivax* malaria, the presence of antibodies to *Pv*MSP-1 protein as well as to the whole parasite was determined in all test sera by ELISA and indirect fluorescent antibody test (IFAT), respectively.

#### Immunogenicity of Recombinant *Pvs*48/45 in BALB/c Mice

Ten randomly selected BALB/c mice (4 weeks old; 20±5g) were divided into two groups. Five experimental mice were immunized with 20 μg of *Pvs*48/45 protein emulsified in Freund Adjuvant and the remaining five mice were immunized with PBS emulsified in Freund Adjuvant 1:1 as a control group. All animals were immunized four times subcutaneously on the base of the tail with a first immunizing dose formulated in Complete Freund Adjuvant (CFA) and the subsequent three doses with a mixture of Incomplete Freund Adjuvant (IFA) and CFA (1:2) in a final volume of 100 μL at 30-day intervals (Fig. 1A). Animals were bled (∼50 μL) prior to each immunization and 30 days after the last immunization. Collected sera were separated and immediately stored at −20°C until use. Specific anti-*Pvs*48/45 antibody titers were determined by ELISA using the recombinant product as described below. Endpoints for mice included body weight, lack of appetite or skin lesions in the immunization site. Body weight was measured before and after each immunization and lack of appetite was daily monitored. At the end of the study, when the humane endpoint were reached, mice were euthanized using CO_2_ inhalation [39] with previous sedation with acepromazine and anesthesia (ketamine/xylazine) by intraperitoneal route to diminish the stress.

**Fig 1:** Immunization Schedule. For: **A.** Mice, animals were immunized four times at 30 days interval with 20 μm of *Pvs*48/45 formulated with Freund Adjuvant. Blood samples were taken on days 0, 30, 60 and 90 for ELISA testing and on day 120 for functional and biological assessing. **B.** Monkeys, two experimental animals were immunized with 50 μg of *Pvs*48/45, and one control group with PBS emulsified in 1:1 with Montanide ISA 51 Adjuvant. Protein was administrated subcutaneously in the back at 20 days intervals, blood samples were taken before each immunization, 15 days after the third immunization and then at 30 days intervals until day 150. EG: Experimental group; CG: Control group; CFA: Freund Complete Adjuvant; IFA: Freund Incomplete Adjuvant; EM: Experimental Monkeys, CM: Control Monkey, ISA 51: Montanide ISA 51 Adjuvant, Prot. *Pvs*48/45 protein.

#### Immunogenicity of Recombinant Pvs48/45 Protein in Primates

From a large group of 20 animals, three (3) male healthy monkeys were randomly selected (4±2 years old; 1,000±200g); IFA and ELISA tests against blood stages and Pvs48/45 respectively, as well as thick smear were performed in order to prove no sero-reactivity with the protein nor gametocytes and discard *Plasmodium* infections. Two of them were immunized with 50 μg of *Pvs*48/45 emulsified in Montanide ISA-51 as adjuvant in final volume of 500 μL. The other one was immunized with 500 μL of a mixture of Montanide ISA-51 and PBS, as a control. All animals received three immunogen booster doses given subcutaneously on their back to minimize pain, at 21-day intervals. Before each immunization,15 days after the last immunization and then at 30 days intervals after day 150 (Fig. 1B). Animals were bled from the femoral vein and sera were separated and stored at -20°C. Antibody titers were measured by ELISA as described below.

#### ELISA Test

96-well plates (Nunc-Immuno Plate, Maxisorp, Roskilde, Denmark) were coated overnight with 50 μL of recombinant *Pvs*48/45 at 1.0 μg/mL and then blocked with 5% skim milk in PBS 1X, 0.05% Tween20 (PBS-T) for 2 hours at room temperature. Test sera diluted 1:200 in 2.5% skim milk in PBS-T were then incubated for 1 hour at 37°C. After washing, the plates were incubated for 1 hour at 37°C with a 1:1,000 or 1:2,000 dilution of alkaline phosphatase-conjugated goat anti-mouse/human IgG antibody (Sigma Chemical Co., St Louis, MO). Cut-off points for ELISA were calculated as three SD above the mean absorbance value at 405 nm of normal mouse sera, normal monkey sera or sera from healthy adult volunteers who had never been exposed to malaria. The results were also expressed as reactivity index (RI) defined as OD values of tested samples divided by the cut-off value.

#### Western Blot Analysis

Infected red blood cells (iRBC) derived from an infected *P*. *vivax* patient were lysed by osmotic shock using water containing a protease inhibitor cocktail followed by three cycles of freezing (-70°C) and thawing (37°C) followed by a sonication cycle at 40°C for 5 min. After centrifugation, the supernatant (SN) was separated and the pellet diluted in 0.1 M Tris-Cl (pH 7.5) and centrifuged at 14,000 rpm for 3 min.

Both antigen SN and pellet were subjected to electrophoresis under reduced conditions using a 12.5% SDS-polyacrylamide gel and electro-transferred to PVDF membranes for 18 hours at 30 v. Membranes were blocked using 3% skim milk for two hours. Serum samples were diluted 1:500 in 1.5% skim milk and incubated for 1 hour. After washing, membranes were incubated with 1:1,000 dilution of alkaline phosphatase-conjugated goat anti-human IgG antibody (Sigma Chemical Co., St Louis, MO) for 1 hour. The reaction was developed with BCIP/NBT alkaline phosphatase substrate (Sigma*Fast*).

#### Indirect Immunofluorescence Antibody Test

*P*. *vivax* enriched iRBCs were used to produce IFAT antigen slides, which were developed as previously described [40]. Serum samples were incubated at 1:10 or 1:20 dilution and labeled with fluorescein isothiocyanate (FITC) conjugated-affinity goat-human IgG antibody at 1:1,500 dilutions. Slides were examined under an epifluorescence microscope and antibody titers were determined as the reciprocal of the end-point dilution that shows positive fluorescence.

#### Transmission-Blocking Assays

TB activity of sera from immunized animals was measured by artificial membrane feeding assays (MFA) as described elsewhere [12]. Briefly, 150 μL iRBCs from a *P*. *vivax* naturally infected patient were washed twice with RPMI 1640 medium (Sigma, St Louis, MO) and diluted in a pool of 150 μL fresh sera prepared by using equal volumes of RPMI medium immunized mice (post-fourth immunization) or monkeys (post-third immunization) to feed ∼100 adult (2–3 day old) *An*. *albimanus* mosquitoes. Post-immunization sera were tested in two-fold serial dilutions up to 1:10 to determine the end point TB activity in monkey plasma collected before immunization and diluted in non-heat inactivated human AB^+^ human serum obtained from the blood bank. The same pool of AB+ normal human sera was used as negative control.

After 30 minutes of feeding, unfed mosquitoes were removed from the cages and fed mosquitoes maintained at 27°C and 80–90% RH. All procedures were performed at 37°C. Seven days after feeding, ∼40 mosquitoes were dissected, midguts were stained with 2% mercurochrome and the number of oocysts per mosquito midgut was counted.

#### Statistical analysis

This is a descriptive study to assess the antigenicity and functional blocking activity of sera and plasma obtained from mice and monkeys immunized with a *Pvs*48/45 recombinant protein by artificial membrane feeding assay. Antibody titers of human sera from different regions and mosquito infectivity outcome were compared by the Fisher’s exact test. Results were considered to be statistically significant when P values were < 0.05.

Two outcomes were determined for the functional TB activity after blood feeding in presence of pool sera from the *Pvs*48/45 immunized BALB/c mice and of plasma from the immunized *Aotus* monkeys: the proportion of infected mosquitoes and the total oocyst counts per mosquito.

## Results

### Bioinformatics Analysis

The primary sequence of *Pvs*48/45 presented 6-Cys domains with 15 Cys residues and the N-terminal signal peptide and the C-terminal GPI anchor which were predicted by the Signal P 3.0 and the GPI-SOM servers. This was demonstrated by multiple alignments between *P*. *vivax Pvs*48/45 with other orthologous proteins including *P*. *berghei* (Pbs48/45), *P*. *yoelii* (Pys48/45), *P*. *chabaudi* (Pcs48/45), *P*. *knowlesi* (Pks48/45) and *P*. *falciparum* (Pfs48/45) (Fig. 2). Additionally, the multiple alignments allowed determination of the identity (70.4%) among P48/45 proteins confirming that P48/45 is highly conserved among *Plasmodium* species. Greater homology was observed with *P*. *knowlesi* (84.0%), whereas for *P*. *falciparum* the homology was 60.8%.

**Fig 2:** Schematic diagram and amino acid sequence alignment of *Pvs*48/45 protein. **A.** Schematic diagram of *Pvs*48/45; boxes in grey represent the three P48/45 domains and the black box at the C-terminal region represents the trans-membrane domain. **B.** Multiple alignments between primary sequences of P48/45 proteins using the software Geneious. Conserved regions are represented in black. Cysteines are shown in blue.

### Cloning, Expression and Purification of *Pvs*48/45

Amplification of the *pvs*48/45 gene without the signal peptide and GPI anchor resulted in the presence of an expected band of ∼1,344 bp in agarose gels (data not shown) that was sub-cloned in a vector for heterologous expression in an *E*. *coli* system with several expression attempts to diminish the probability of generating antibacterial toxic products. Affinity chromatography allowed purification of a protein of ∼60kDa in SDS-PAGE, which corresponds to the predicted weight of the protein (65.4 kDa). This includes the 6-His tag under reducing conditions (Fig. 3A).

**Fig 3:** *Pvs*48/45 protein expression in *E*. *coli*. **A.** 10% SDS-PAGE stained with Coomasie blue. Lane 1, molecular weight marker; lane 2, un-induced cells total extract; lane 3, purified *Pvs*48/45 under reducing conditions (10mM β-mercaptoethanol). **B.** Western blot of *Pvs*48/45. Lane 1, molecular weight marker; Lane 2, un-induced cells total extract under reducing conditions (10mM β-mercaptoethanol). Lane 3, *Pvs*48/45 revealed against anti-His antibody; Lane 4, *Pvs*48/45 revealed against hyper-immune monkey sera. Arrows indicate the expected weight. **C.** Mass spectrum of *Pvs*48/45.

The purified protein was recognized by the primary anti-His antibody as well as by sera from hyper-immune monkeys upon development with NBT/BCIP (Fig. 3B). The yield was ∼1mg/L of bacterial culture. To identify the recombinant protein, the purified product was subjected to mass spectrometry analysis (LC-MS/MS). Database analysis identified three unique peptides derived from *Pvs*48/45 with a high score in the MASCOT server (Table 1). This result was confirmed by cleaning the spectra using Scaffold software, which yields a 100% probability for the identification of *Pv*s48/45. The correct molecular weight was confirmed by mass spectrometry at 65.8 kDa (Fig. 3C).

**Table 1:** Observed values of tryptic peptides from the *Pvs*48/45 by MS/MS.

Peptide	Sequence	Scaffold Prob	Mascot Ion score	Mascot Identity score	Observed	Charge	Delta Da
1	VALVQVNVLK	99%	35.2	31.2	542.12	2	0.0029
2	IFGLVGSIPK	99%	31.6	28.3	541.85	2	0.0039
3	ITSINLTK	99%	29.5	25.0	515.82	2	0.0037

### *Pvs*48/45 Antigenicity

Specific anti-*Pvs*48/45 antibody responses were found in 19/30 (63.3%) of the human serum samples tested with reactivity ranging from RI 1.04 to 2.87. Reactivity to *Pv*MSP-1 (r200L fragment) was found in 15/30 (50%) samples and 33.3% presented reactivity to both antigens (Table 2). Although the number of sera samples analyzed was limited, a more frequent recognition was observed in samples collected from Tumaco, Buenaventura and Chocó in the Pacific regions (13/15 or 86.6%) compared to those collected in Tierralta in the Caribbean region (6/15 or 40%) with a significant difference between the two regions (p = 0.021 by a Fisher’s exact test). Additionally, the frequency of reactivity to *Pvs*48/45 appeared to be age-dependent (Table 2).

**Table 2:** Antigenicity of r*Pvs*48/45 protein in human serum samples from Colombia.

Age range	Responders % (positive samples/total samples)		Reactivity index range*
	MSP-1	*Pvs*48/45	*Pvs*48/45
0–10	20.0 (1/5)	40.0 (2/5)	1.04–1.13
11–17	33.3 (2/6)	50.0 (3/6)	1.25–2.22
18–30	85.7 (6/7)	57.1 (4/7)	1.30–2.87
30–60	50.0 (6/12)	83.3 (10/12)	1.08–1.93
**Positivity by Region**			
Caribbean	46.6 (7/15)	40.0 (6/15)	1.04–2.22
Pacific	53.3 (8/15)	86.6 (13/15)	1.08–2.87

* Were analyzed only samples with RI>1.0

### *Pvs*48/45 Immunogenicity

All mice immunized with the recombinant protein developed high titers of antibodies specific to the r*Pvs*48/45 protein and all seroconverted after the first dose. A boosting effect was observed with the two subsequent immunizations at 30 and 60 days. ELISA titers increased to 3x10^6^ after the third immunization on day 60 (Fig. 4A).

**Fig 4:** Immune responses to r*Pvs*48/45. In **A.** BALB/c mice. Serum samples were collected pre-immunization on day 0 and post-immunization on days 30, 60, 90 and 150 and **B. *Aotus lemurinus griseimembra***. Kinetics of antibody titers in *Aotus* during immunization and follow-up period. Experimental monkeys immunized with 50 μg r*Pvs*48/45 formulated in Montanide ISA-51; Control monkey immunized with a mixture of Montanide ISA-51 and PBS 1X. Titers correspond to the last dilution of the test sera in which OD_405_ values were above that of the cut-off. Cut-off value were defined as pooled naïve mouse or monkey sera, OD_405_ plus 3SD. Serum samples were tested at two-fold serial dilutions (1x10^2^–2x10^5^); a pool serum from naïve mice was used as negative control.

Likewise, the two *Aotus* monkeys immunized with the r*Pvs*48/45 showed antibody titers ranging between 1.6 x10^4^ and 3.2 x 10^4^. One of the *Aotus* monkeys seroconverted after the first dose, whereas the other one needed two doses to seroconvert. The animals reached the higher titers after three immunizations and antibodies remained detectable in both animals for more than five months of follow-up after the last immunization (Fig. 4B). Control monkey did not seroconvert anytime during the experiment. Neither serious adverse events nor side effect were observed after immunization and all levels of hematological, liver and kidney function parameters remained at baseline values.

### Recognition of the Parasite Protein in WB and IFAT

Sera from immunized monkeys recognized the protein in WB assays performed using as antigen the whole parasites derived from a *P*. *vivax* infected patient under reducing and non-reducing conditions. A distinct band of ∼60 kDa was observed under reducing conditions when the iRBCs lysis-SN was analyzed. Non-reduced protein showed less electrophoretic mobility. Recognition of pellet extracts was poor (Fig. 5A and 5B). In addition, IFAT using parasite preparations containing gametocytes indicated the strong reactivity of all sera samples tested (Fig. 5C).

**Fig 5:** Recognition of parasite *Pvs*48/45 protein by sera of immunized monkeys. **A)** Western blot assay using antigen extracted from pellet after iRBCs lysis in reduced conditions (β-mercaptoethanol). Lane 1, antigen (non-diluted); lane 2, antigen 1:2 diluted; lane 3, antigen 1:4 diluted. **B)** Western blot assay using antigen extracted from supernatant after iRBCs lysis in reduced conditions (β-mercaptoethanol). Lane 1, antigen (non-diluted); lane 2, antigen 1:2 diluted; lane 3, antigen 1:4 diluted. Triangles indicate increased concentration. **C)** Monkey IgG was reactive with *Pvs*48/45 on acetone-fixed smears of sexual blood stages of *P*. *vivax* with monkey sera containing antibodies to r*Pvs*48/45. From left to right: parasite in light (left), parasite in epifluorescence (right).

### Functional Activity of Anti *Pvs*48/45 Antibodies

Functional activity of mouse sera tested using three different *P*. *vivax* isolates in independent MFAs indicated strong reproducible TB activity. A pool of sera collected four weeks after the last mouse immunization displayed full inhibition of parasite transmission to mosquitoes in MFA. Likewise, a pool of sera from monkeys after the last immunization showed functional TB activity in three independent MFAs, in which full TB activity was observed. Significant differences were observed between this TB activity and the pre-immunization and AB sera used as control (P value < 0.0001 by Fisher's exact test) (Table 3). Blocking effects was maintained in monkey plasma diluted up to 1:8 with a TB activity of 52%.

**Table 3:** Transmission blocking activity of sera from immunized animals.

Type of sera	Assay No.	Negative control (naive human sera AB+)		Experimental sera	
		% Infection	Oocyst Mean (SEM)	% Infection	Oocyst Mean (SEM)
BALB/c mice	1	75 (30/40)	16.2 (3.4)	0 (0/40)	0
	2	67,6 (25/37)	1.4 (0.2)	0 (0/30)	0
	3	43,3 (13/30)	10.5 (3.8)	0 (0/30)	0
*Aotus* monkeys	1	50 (25/50)	2.9 (0.9)	0 (0/40)	0
	2	52 (26/50)	1.6 (0.5)	0 (0/40)	0

Numbers within parentheses indicate total number of infected mosquitoes/total number of mosquitoes dissected for each MFA.

## Discussion

We report the functional TB activity of a *Pv*s48/45 recombinant protein produced in *E*. *coli* using a harmonized sequence, which leads to high yields of a properly folded protein and conserved conformational epitopes. Epitopes with conformation similar to the native protein were indirectly determined to be present in the recombinant product by protein reactivity with antibodies elicited by both the natural exposure to *P*. *vivax* malaria in endemic areas as well as by the recognition of parasite proteins by antibodies produced through experimental animal immunizations with the *Pvs*48/45 recombinant protein. Even more interesting is the fact that anti-*Pv*s48/45 antibodies produced by immunized mice and monkeys efficiently blocked parasite transmission to *An*. *albimanus* mosquitoes in *ex-vivo* MFA.

Although heterologous protein production in *E*. *coli* has become a routine method for proteins of different characteristics, the expression of soluble and functional malaria proteins in bacteria still represents a challenge due to considerations of cost, speed, ease of use and genetic manipulation [41]. Furthermore, it frequently results in a lack of expression, poor protein solubility due to the aggregation of the recombinant product in inclusion bodies, and in cellular toxicity. Several *Plasmodium* genome features are thought to hinder optimal expression of malarial proteins. These features are: 1) the *P*. *falciparum* genome exhibits an unusually high content of adenine and thymine (AT = 80%); 2) *P*. *falciparum* proteins are larger than their homologues in others malaria species; and 3) *Plasmodium* parasites display post-translational modifications that are unique to this parasite species [42]. Although in many aspects the *P*. *vivax* genome is similar to that of *P*. *falciparum*, *P*. *vivax* (Salvador 1 strain) contains AT-rich chromosome ends and has a telomere-distal regions which consists of GC-rich sequences [43,44]. This results in low transcription efficiency in *E*. *coli*, *which* affects the protein yield in bacteria. In addition, the heterologous expression of *Plasmodium* proteins has the limitation of incorrect folding of the protein in the non-natural host, slowing the progress of antimalarial vaccine development.

To overcome these disadvantages, many strategies have been designed [45]. As such, *E*. *coli* remains as the preferred host for heterologous protein expression, including the functional expression of soluble *Plasmodium* proteins [46]. In this study, we designed a strategy to express the recombinant protein using a full codon harmonization approach followed by the expression using the pET32a expression vector which increases solubility by adding a thioredoxin domain to the protein. This feature makes the vector useful for *Pvs*48/45 expression.

Confirmation of the high antigenicity of the r*Pvs48*/45 is a significant finding as it confirms that there is production of anti-*Pvs*48/45 antibodies upon natural exposure to the parasite infection despite the fact that gametocyte growth and maturation occurs intracellularly. However, this may be explained by the fact that the gametocytes eventually die inside the circulation of the vertebrate host before being transferred to the mosquito, thereby becoming available for priming the immune system and eliciting specific antibodies; additionally, gametocyte-iRBC may release intracellular antigens into the host circulation. Reactivity of natural antibodies with the recombinant protein is also an indication that at least some of the domains containing immune epitopes are present in the recombinant protein in a proper conformation. This includes the possibility that some epitopes may be linear. Moreover, the presence of epitopes with similar conformation as in the native protein was indirectly confirmed by recognition of the parasite protein by antibodies raised through immunization of experimental animals (mice and primates) with the recombinant protein. Even more interesting is the fact that anti-*Pvs*48/45 antibodies produced by immunized animals efficiently and consistently blocked parasite transmission to *An*. *albimanus* mosquitoes in *ex-vivo* MFA.

Although numerous questions remain to be answered about this protein and its role in TB under natural conditions, this r*Pvs48*/45 represents a valuable reagent for further study of the importance of naturally-elicited antibodies in endemic areas i.e. the TB efficacy of purified human antibodies. It also allows better characterization of immune mechanisms, e.g. the definition of relevant protein domains; the influence of complement in affecting the TB potency of naturally-elicited antibodies; and the protein’s capacity to induce protective T-cell responses. More importantly, primate studies would allow the definition of the potential prime-boost effect of r*Pvs48*/45; gametocytes are expected to be able to boost the antibody responses elicited artificially by immunization. Likewise, it is probable that r*Pvs48*/45 is able to induce boosting of naturally-existing antibodies in endemic populations. It is encouraging that antibody titers elicited by the vaccine formulation used here remained high for at least six months. Given the availability of r*Pvs48*/45, the primate model, and the MFA system, further studies are warranted to determine these different features using the primate model as well as the role of naturally acquired antibodies.

## Supporting Information

S1 ARRIVE Checklist ARRIVE Checklist Recombinant Pvs4845 antigen expressed in E. coli. (PDF)
